The article "Targeting Molecular Mediators of Ferroptosis and Oxidative Stress for Neurological Disorders" was published in 2022. Journal: Oxid Med Cell Longev.

# Targeting Molecular Mediators of Ferroptosis and Oxidative Stress for Neurological Disorders

**DOI:** 10.1155/2022/3999083

**Published:** 2022-07-22

**Authors:** Jing Li, Bowen Jia, Ying Cheng, Yiting Song, Qianqian Li, Chengliang Luo

**Affiliations:** ^1^Department of Forensic Medicine, School of Basic Medicine and Biological Sciences, Soochow University, Suzhou 215123, China; ^2^School of Forensic Medicine, Wannan Medical College, Wuhu 241002, China

## Abstract

With the acceleration of population aging, nervous system diseases including Alzheimer's disease (AD), Parkinson's disease (PD), Huntington's disease (HD), anxiety, depression, stroke, and traumatic brain injury (TBI) have become a huge burden on families and society. The mechanism of neurological disorders is complex, which also lacks effective treatment, so relevant research is required to solve these problems urgently. Given that oxidative stress-induced lipid peroxidation eventually leads to ferroptosis, both oxidative stress and ferroptosis are important mechanisms causing neurological disorders, targeting mediators of oxidative stress and ferroptosis have become a hot research direction at present. Our review provides a current view of the mechanisms underlying ferroptosis and oxidative stress participate in neurological disorders, the potential application of molecular mediators targeting ferroptosis and oxidative stress in neurological disorders. The target of molecular mediators or agents of oxidative stress and ferroptosis associated with neurological disorders, such as reactive oxygen species (ROS), nuclear factor erythroid 2–related factor-antioxidant response element (Nrf2-ARE), n-acetylcysteine (NAC), Fe^2+^, NADPH, and its oxidases NOX, has been described in this article. Given that oxidative stress-induced ferroptosis plays a pivotal role in neurological disorders, further research on the mechanisms of ferroptosis caused by oxidative stress will help provide new targets for the treatment of neurological disorders.

## 1. Introduction

As a novel mode of regulated cell death (RCD), ferroptosis was firstly proposed by Dixon in 2012 [1]. Ferroptosis is an iron-dependent and nonapoptotic cell death mode, which is caused by excessive accumulation of ROS and imbalance of cell lipid oxide metabolism. In 2018, the Nomenclature Committee on Cell Death (NCCD) advised defining ferroptosis as RCD caused by oxidative stress in the cell microenvironment which can be regulated by glutathione peroxidase 4 (GPX4). Moreover, ferroptosis can be inhibited by iron chelators, iron intake inhibitors, and lipophilic antioxidants [2, 3]. Recent studies have shown that ferroptosis is obviously different from traditional programmed cell death. It has distinctive morphological features and biochemical features [4], such as morphological changes of mitochondrial, accumulation of iron, and lipid reactive oxygen species (ROS). At present, it is believed that the main cause of ferroptosis to cell death is the inactivation of the cellular antioxidant system, which includes the inhibition of cystine/glutamate antiporter system (system Xc^–^) and GPX4, disrupted iron homeostasis, and lipid peroxidation. Ultimately, the decrease of antioxidant capacity and the accumulation of intracellular lipid ROS lead to oxidative cell death [5].

The article "Targeting Molecular Mediators of Ferroptosis and Oxidative Stress for Neurological Disorders" was published in 2022. Journal: Oxid Med Cell Longev.

Although there are many studies about ferroptosis, the mechanism of ferroptosis is not clear yet. Ferroptosis was identified to involve in oxidative stress-induced cell death [6]. During the process of ferroptosis, cellular over-accumulation of ROS eventually generates oxidative stress and cell death. According to current research, the possible mechanisms of ferroptosis include oxidative stress, lipid peroxidation, iron metabolism, and other mechanisms to be explored. The process of oxidative stress in ferroptosis is complex that is regulated by a variety of regulatory factors.

Neurological disorders have become the major leading cause of disability and the second leading cause of death worldwide [7]. Over the past few decades, due to the lack of effective precaution and treatment, the mortality and the disabled owing to neurological diseases have increased, particularly in low-income and middle-income countries [8]. The death and disability caused by neurological disorders have caused a huge burden on families and countries. Meanwhile, it has become a serious social problem. In order to alleviate the burden, there are increasing studies on how to treat or prevent the process of neurological disorders.

Mounting evidence has shown that oxidative stress-induced ferroptosis plays a significant role in neurological disorders [3]. Oxidative stress is both an important process of ferroptosis and the pathogenesis of neurological disorders. Hence, oxidative stress has become a critical linking between ferroptosis and neurological disorders. Up to now, the inhibitors and activators of ferroptosis [9–14], as well as other involved signaling pathways [15–17], have been widely studied. Furthermore, the mediators of oxidative stress might become a potential therapeutic target for the treatment of neurological disorders by regulating the process of ferroptosis. In this review, we will briefly summarize the mechanisms of ferroptosis, and highlight the role of targeting molecular mediators of oxidative stress in neurological disorders, so as to provide an option for the therapeutic application of ferroptosis in neurological disorders.

The article "Targeting Molecular Mediators of Ferroptosis and Oxidative Stress for Neurological Disorders" was published in 2022. Journal: Oxid Med Cell Longev.

## 2. The Mechanism of Ferroptosis

Ferroptosis is a unique kind of nonapoptotic-regulated cell death, which is distinct from apoptosis, autophagy, and necrosis in morphology, biochemistry, and genetics. Iron metabolism and lipid peroxidation are two essential events in ferroptosis [2]. Additionally, system Xc^−^ and GPX4 are considered to be the primary signaling pathways [18]. Here, we summarize the main mechanisms involved in the process of ferroptosis, such as oxidative stress, lipid peroxidation, iron metabolism, and the signaling pathways (Figure 1).

### 2.1. Oxidative Stress in Ferroptosis

Oxidative stress was formulated in 1985 [19], which is an important cause leading to neurological disorders that mainly arise from the imbalance between depletion of antioxidants and production of peroxides [20]. Ferroptosis is a unique, oxidative stress-induced cell death pathway characterized by glutathione depletion and lipid peroxidation. Based on current research, ferroptosis can be regulated by system Xc^–^ [21]. System Xc^–^ can exchange glutamate and cystine inside and outside of the cell. Glutathione is an important free radical scavenger and antioxidant in vivo, which can be categorized as either reduced (GSH) or oxidized (GSSG). Intracellular cystine can be converted into reduced GSH by a series of biochemical reactions. GPX4 is a member of the glutathione peroxidase family which can convert GSH to GSSG, and GSH/GSSG constitutes an antioxidant system and provides reducing equivalents to eliminate oxidative species [22]. GPX4 is a redox enzyme and can also inhibit ferroptosis by decreasing the level of lipid peroxides. GPX4 plays a crucial role in reducing reactive aldehydes (PUFAs-OOH) to their alcohol form (PUFAs-OH) which can reduce the content of ROS [18].

ROS are some of the most common oxidants in cells. ROS includes superoxide (O_2_^−^•), hydrogen peroxide (H_2_O_2_), lipid peroxides (ROOH), or the corresponding hydroxyl (HO•) and peroxyl radicals (ROO•) [23]. Accumulation of ROS can lead to oxidative stress, causing oxidative stress-induced lipid peroxidation. What is worse, lipid peroxidation may further generate ROS or degrade into reactive compounds capable of crosslinking DNA and proteins [24]. Oxidative stress-induced lipid peroxidation eventually leads to ferroptosis. Meanwhile, ferroptosis can be induced by oxidative stress directly (Figure 1).

### 2.2. Iron Metabolism in Ferroptosis

Metabolism is essential for the biochemical process in cells and goes awry in many diseases. Iron metabolism is an important mechanism of ferroptosis [2]. Iron is a significant trace element in the body [25]. Abnormal distribution and content of iron in the body can affect the normal physiological processes. Fe^2+^ is absorbed by the intestine or degraded by erythrocyte and then can be oxidized to Fe^3+^ by ceruloplasmin [26]. Fe^3+^ can combine with transferrin (Tf) on cytomembrane to form Fe^3+^-Tf, which can be endocytosed into cells to form a complex with membrane protein TF receptor (Tfr) [26]. The complex enters the endosome and is divided into TF-TFR and Fe^3+^ [26]. Fe^3+^ is then reduced to Fe^2+^ by the six-transmembrane epithelial antigen of the prostate 3 (STEAP3), and Fe^2+^ is stored in the unstable iron pool (LIP) and ferritin [26]. Nevertheless, under pathological conditions, iron homeostasis is destroyed, and the overwhelming production of Fe^2+^ exceeds the limit, breaking cell homeostasis [27]. Excess Fe^2+^ can combine with H_2_O_2_, reducing H_2_O_2_ to hydroxyl radical (OH·) by Fenton reaction [28, 29], which was first described by Fenton [30], who in 1894 reported on the oxidation of malic acid by hydrogen peroxide in the presence of ferrous ions.

The article "Targeting Molecular Mediators of Ferroptosis and Oxidative Stress for Neurological Disorders" was published in 2022. Journal: Oxid Med Cell Longev.

### 2.3. Role of Mitochondria in Ferroptosis

Mitochondria, through the tricarboxylic acid cycle (TCA) and electron transport chain (ETC) activity, are the principal sources of cellular energy production [31]. Meanwhile, ROS can be produced during the process of TCA which is an important cause of ferroptosis-induced lipid peroxides [32]. In addition, mitochondrial morphological changes are considered to be an important basis for the diagnosis of ferroptosis [1]. The change of mitochondrial membrane potential is also an important discovery in the study of ferroptosis [33, 34]. To date, abnormal mitochondrial architecture including mitochondrial fragmentation, rupture of mitochondrial outer membrane, and mitochondrial shrinkage, as well as vanished mitochondrial cristae, is regarded as the typical morphological characteristic of ferroptosis [1]. In summary, mitochondria play a significant role in ferroptosis [35], and molecular research targeting mitochondria is of great significance to intervene in the development of ferroptosis (Figure 1).

### 2.4. Other Mechanisms

As a novel form of cell death, the mechanism of ferroptosis is complex. Ferroptosis is regulated by numerous pathways and implicated in many diseases. In addition to the mechanisms mentioned above, there are other possible mechanisms which have been proposed, such as the antioxidant mechanisms which include GPX4 pathway [36], FSP1 pathway [37], and other pathways. FSP1-NADPH-CoQ pathway [38] and nuclear factor erythroid 2-related factor 2 (Nrf2) pathway are potential regulatory pathways of ferroptosis [39]. Hence, the mechanism of ferroptosis remains to be explored.

The article "Targeting Molecular Mediators of Ferroptosis and Oxidative Stress for Neurological Disorders" was published in 2022. Journal: Oxid Med Cell Longev.

## 3. Ferroptosis in Neurological Disorders

In recent years, the incidence of neurological disorders increases substantially. Because of the lack of effective treatment, sequelae caused by neurological disorders have brought an enormous burden on society. Ferroptosis has been proved to be closely related to the occurrence and development of various neurological disorders [40–43]. Therefore, figuring out the role of ferroptosis in neurological disorders will provide an important basis for the treatment of diseases (Figure 1, Table 1).

### 3.1. Ferroptosis in Parkinson's Disease

Parkinson's disease (PD), also called paralysis agitans, is the second most common neurodegenerative disorder worldwide. It is typical of neuronal death in the substantia nigra pars compacta (SNpc), which adjusts motor function. PD causes clinical symptoms such as resting tremor, rigidity, bradykinesia, postural instability, and other motor symptoms [44–46]. However, its basic mechanism is not completely clear. Currently therapeutic arsenal mainly includes the application of the dopamine precursor levodopa (L-DOPA), dopamine metabolism inhibitors, and dopamine agonists [33], which only offer symptomatic relief. There still are not effective treatments for PD, so novel targets to improve therapeutic and diagnostic methods for PD patients are urgently needed. Iron is considered to be an important target of neurodegenerative diseases. Besides, iron metabolism is closely related to the pathogenesis of neurodegenerative diseases [34, 47]. Researchers found that patients with PD suffered from GSH depletion, ROS elevation, and lipid peroxidation [48–50]. Ferritin heavy chain 1 (FTH1), a main iron storage protein, can affect intracellular iron metabolism and then trigger ferroptosis. As an important ferroptosis-related protein, FTH1 is differentially expressed in rats with PD compared with normal rats. Overexpression of *FTH1* can reduce the effect of ferroptosis in PD-related cells [51]. These findings indicate that ferroptosis may be used as a therapeutic target for PD [52, 53]. Neuroimaging and postmortem examination report that much iron accumulation in substantia nigra (SN) results in an increase in iron content in the residual dopaminergic neurons [54]. *α*-Synuclein causes iron cytotoxicity by acting on mitochondria in the neurodegeneration of PD. A study found that cyclosporine A, a blocker of mitochondrial permeability transition pore (mPTP), could prevent iron-induced mitochondrial damage and cell death. Furthermore, knocking down *α*-synuclein expression by siRNA can play a similar role [55]. *α*-Synuclein is the main component of Lewy bodies and is abundantly expressed in the nervous system, which is strongly related to PD's pathophysiology [56]. Besides, it has been recently shown that *α*-synuclein causes lipid peroxidation by producing ROS, leading to increased calcium influx and consequent cell death [57]. Ferroptosis inhibitors like ferrostatin or iron chelators [58] can inhibit cell death caused by the above method, supporting the hypothesis that ferroptosis participates in this process and may harbor therapeutic potential. Studies have also shown that ferroptosis occurs earlier than apoptosis in the development of PD and ferric ammonium citrate (FAC)-induced ferroptosis was dependent on p53, not MAPK signaling pathway [54].

The article "Targeting Molecular Mediators of Ferroptosis and Oxidative Stress for Neurological Disorders" was published in 2022. Journal: Oxid Med Cell Longev.

### 3.2. Ferroptosis in Alzheimer's Disease

Alzheimer's disease (AD) is one of the most common neurodegenerative diseases worldwide. Pathological features of AD include cerebral atrophy, intraneuronal accumulation of hyperphosphorylated tau in neurofibrillary tangles, extracellular deposition of amyloid-*β* peptide in senile plaques, oxidative stress, chronic inflammation, and loss of neurons and synapses [59]. There is evidence that iron excess and homeostasis disorder can lead to neurodegeneration of AD [60, 61]. The increase of brain iron content in patients with AD has been confirmed in many studies [62–67]. When brain iron regulation in AD patients is disturbed, excess Fe^2+^ can not only produce hydroxyl radicals in Fenton reaction but also induce neuroinflammation, resulting in oxidative stress and neurodegeneration mediated by ferroptosis [68–72]. The research found that the increase of ferritin light chain (FTL) is related to the decrease of GPX4 level in AD which indicates that dysfunctional ferritin will reduce the antioxidant capacity of brain and the level of glutathione will decrease in AD patients [73]. Increased light subunit (xCT) expression in cells of patients with AD [74] and xCT can be upregulated by Nrf2 [75, 76]. Furthermore, mice with a conditional deletion of GPX4 show cognitive impairment and hippocampal degeneration similar to patients with AD and have the neurodegenerative characteristics of ferroptosis. Simultaneously, these symptoms can be improved by ferroptosis inhibitors [77], which provide a basis for the association between AD and ferroptosis. Recently, researchers observed that tau can stabilize ferroportin (FPN1) which is the only iron export channel found in mammalian cells [78, 79]. FPN decreased significantly in the brain tissue of AD patients. According to MMSE (mini-mental state examination) scores, FPN is involved in the cognitive impairment and brain atrophy of AD [80]. In patients with AD and a mouse model of AD, NADPH oxidases 4 (NOX4) causes lipid peroxidation and promotes ferroptosis of astrocytes via the damage of mitochondrial metabolism in AD [81]. Bhatia et al. [82] summarized a variety of multitarget targeted ligands with iron chelation properties, which is potentially useful in AD. Ashraf et al. [83] summarized the clinical cases involving iron chelators, antioxidants, NAC, and selenium in the treatment of AD and provided a feasible basis for the treatment of AD. These studies have shown that ferroptosis plays an important role in AD, in which a variety of regulatory factors are involved, and provide many potential therapeutic targets for the treatment of AD.

The article "Targeting Molecular Mediators of Ferroptosis and Oxidative Stress for Neurological Disorders" was published in 2022. Journal: Oxid Med Cell Longev.

### 3.3. Ferroptosis in Huntington's Disease

Huntington's disease (HD) is an autosomal dominant, late-onset, and fatal neurodegenerative disorder [84], which is caused by an abnormal CAG repeat in the huntingtin gene [85]. It is characterized by highly selective striatal injury, leading to dance-like movement, progressive dementia, and dystonia. In 2001, Pigeon et al. [86] first identified the association between hepcidin and iron homeostasis. Studies found that hepcidin could promote ferroptosis through iron metabolism [87] and could prevent erastin-induced ferroptosis by degrading Fpn [88]. Qian et al. [89] summarized the therapeutic potential of hepcidin in neurodegenerative diseases, including HD, indicating that there is a link between ferroptosis and HD. A study found that there is an accumulation of toxic iron in neurons of mouse model with HD and the symptoms of HD can be alleviated by deferoxamine, indicating that the accumulation of iron may contribute to the neurodegenerative process [90]. Studies have shown that HD patients will cause oxidative stress and neurotoxicity to neurons in the striatum, resulting in neuronal death, and eventually leading to motor and cognitive impairment [91]. HD patients have shown higher levels of plasma lipid peroxidation and lower GSH levels [92]. Oxidative stress and lipid peroxidation are important mechanisms leading to ferroptosis. In 2017, Cardoso et al. [93] proposed that as a key factor in regulating ferroptosis, GPX4 could provide protective mechanisms against neurodegeneration. Skouta et al. [94] found that ferroptosis inhibitor Fer-1 and its derivatives can prevent cell death in HD brain slice model. Mi et al. [85] summarized the evidence of ferroptosis involved in HD in different animal models or human patients. It revealed the close connection between ferroptosis and HD which would provide an important potential target for the treatment of HD.

### 3.4. Ferroptosis in Anxiety and Depression

With the development of society, the incidence rate of anxiety and depression is increasing year by year. The research on the mechanism and the treatment of anxiety and depression have also attracted extensive attention. Jiao et al. [95] found that the contents of total iron and ferrous ion in the hippocampus of chronic unpredictable mild stress (CUMS) model mice increased, and GPX4, FTH1, ACSl4, and COX-2 also changed significantly, which proved the evidence of ferroptosis in the hippocampus of the depression mouse model. Previous research reported that sodium hydrosulfide (NaHS) can alleviate the depressive and anxiety-like behaviors induced by type 1 diabetes mellitus (T1DM) [96]. Wang et al. [97] revealed that NaHS reduced ferroptosis in the prefrontal cortex (PFC) of the T1DM mouse model by reducing iron deposition and oxidative stress, increasing the expression of GPX4 and SLC7A11, thus alleviating the anxiety-like and depression-like behavior of the mouse model with T1DM. Moreover, there is increasing evidence that oxidative stress has close contact with anxiety and depression [98, 99]. As a free radical scavenger [100], Edaravone (3-methyl-1-phenyl-2-pyrazolin-5-one, EDA) can improve depression and anxiety-like behavior, as well as inhibit oxidative stress and neuroinflammation in a mouse model of depression, and knocking down of GPX4 expression in CSDs mouse model can inhibit the therapeutic effect of EDA on depression and anxiety [101]. The study has shown that GPX4 can affect the role of EDA in mouse models of anxiety and depression, which suggests that GPX4-mediated ferroptosis may be a potential mechanism affecting anxiety and depression.

The article "Targeting Molecular Mediators of Ferroptosis and Oxidative Stress for Neurological Disorders" was published in 2022. Journal: Oxid Med Cell Longev.

### 3.5. Ferroptosis in Stroke

Stroke is mainly divided into ischemic stroke and intracerebral hemorrhage (ICH) stroke, the former accounting for a higher proportion [102]. Zhang et al. [103] summarized the multiple roles of ferroptosis in stroke. Jin et al. [104] reviewed some neuroprotectants that show protective effects in stroke models. These substances have been recently validated as ferroptosis inhibitors. These researches indicate that ferroptosis plays a key role in the progression and toxicity of stroke. Chen et al. [105] analyzed and identified ferroptosis-related differentially expressed genes (DEGs) in ischemic stroke by bioinformatics, which provided more evidence for the important role of ferroptosis in ischemic stroke. NAC is considered as a potential therapeutic agent of ferroptosis. Recently, studies have found that NAC can reduce neuronal death and improve functional recovery in mouse models with ICH by inhibiting ferroptosis [106]. Clinical trials and experimental studies have reported that treatment with natural compounds could reduce oxidative stress in ischemic stroke. [107]. Therefore, reducing the production of ROS during reperfusion is the key to the treatment of ischemic stroke. Guan et al. found that natural product carvacrol can increase the expression of GPX4 to inhibit ferroptosis, protecting the cognitive function of mice with ischemia-reperfusion injury [108]. In addition, Cui et al. revealed that ACSL4 can exacerbate ischemic stroke by promoting ferroptosis-induced brain injury and neuroinflammation [109]. The incidence rate of ICH is low, but the deformity and mortality rates are significantly higher than ischemic stroke [110]. ICH can lead to the rupture of blood vessels in the brain and release red blood cells to produce a large amount of free iron and ROS, which result in oxidative stress and ultimately neuronal damage [111]. Iron chelator deferoxamine (DFO) can effectively alleviate ICH-induced neuronal injury in mice [112], which also provides evidence for the above process. The same characteristics of ferroptosis were observed in the animal model of ICH [113]. Furthermore, selenium can drive adaptive transcription against ferroptosis to protect neurons and provide direction for the treatment of stroke [114].

The article "Targeting Molecular Mediators of Ferroptosis and Oxidative Stress for Neurological Disorders" was published in 2022. Journal: Oxid Med Cell Longev.

### 3.6. Ferroptosis in TBI

As one of the acute central nervous system (CNS) trauma [115], traumatic brain injury (TBI) is a major cause of death and disability worldwide [116]. Owing to the difficulty of treatment and serious sequelae, TBI has always been a huge problem in the medical field and caused a huge burden on families and society [41]. Analyzing the mouse TBI model [117] and clinical cases with TBI [118], abnormal regulation of ferroptosis after TBI was found both in experimental model and clinical cases. Interestingly, Xie et al. found that the content of iron in damaged cortical cells increased, the function of iron metabolism was impaired, lipid ROS accumulation was increased, and mitochondrial atrophy was enhanced. The above symptoms can be alleviated by intraventricular administration of ferroptosis inhibitor Fer-1 in a mouse model with TBI [119], which proves that ferroptosis is one of the causes of TBI. Previous studies have shown that mir-212-5p is highly expressed in the brain [120] and is associated with a variety of neurological diseases [77, 119, 121, 122]. The use of mir-212-5p in the CCI mouse model can target PTGS2 to reduce ferroptosis and protect the brain [123]. Moreover, Cheng et al. [124] found that the use of iron uptake inhibitor ferristatin II in mouse model with TBI can inhibit the formation of iron proteasomes and alleviate TBI injury in brain. For a long time, due to the lack of clear understanding, the treatment of TBI is very difficult. These studies provide a potential theoretical basis for the treatment of TBI.

The article "Targeting Molecular Mediators of Ferroptosis and Oxidative Stress for Neurological Disorders" was published in 2022. Journal: Oxid Med Cell Longev.

## 4. Mediators of Oxidative Stress in Neurological Disorders

Oxidative stress can spread, which aggravates the production of ROS. Due to the high oxygen demand and high energy demand of the brain, but its antioxidant capacity is weak, it is more vulnerable to oxidative stress [125], which will lead to various neurological diseases. Therefore, inhibiting or weakening oxidative stress might effectively reduce the damage to the nervous system. Studies for targeting molecular mediators of oxidative stress are considerable and will provide effective treatment for neurological disorders (Figure 2).

### 4.1. Nrf2-ARE-Mediated Oxidative Stress

Nuclear factor erythroid 2–related factor (Nrf2) is a transcription factor belonging to the basic leucine zipper (bZIP) transcription factor family that can participate in the regulation of oxidative stress. The antioxidant capacity of Nrf2 works by inducing glutathione biosynthesis [126]. Studies found that Nrf2 can play a neuroprotective role in central nervous system (CNS) diseases [127–129]. In addition to the transcriptional regulation of Nrf2, current hot research directions for the activity of Nrf2 are Kelch-like ECH-associated protein 1 (Keap1)/Nrf2/antioxidant response element (ARE) pathway. Keap1/Nrf2/ARE can be divided into two parts, one in the cytoplasm and the other in the nucleus. Normally, Keap1 and Nrf2 bind in the cytoplasm and are in an inactive state. If they are not activated all the time, Nrf2 will be ubiquitinated and then degraded. Under certain stimulation, the binding of keap1-nrf2 will be unstable. Nrf2 will be released, transferred to the nucleus, combined with ARE, activate the transcription of downstream genes, and then translate a series of related proteins, which can induce various antioxidant enzymes, including heme oxygenase 1 (HO-1), NAD (P) H: quinone oxidoreductase 1 (NQO1), superoxide dismutase (SOD), glutathione peroxidase (GPX), and catalase (CAT). These enzymes can play physiological functions [130]. Targeted regulators of Nrf2 are of great significance in the treatment of oxidative stress-induced injury in neurological disorders. Nrf2 plays a neuroprotective role by regulating the antioxidant system of cells. The regulation will have an impact on glutathione (GSH), thioredoxin (TXN), NADPH, and various other ROS-related enzymes [131, 132].

Keap1/Nrf2/ARE pathway has been proved to be an important antioxidant target. Keap1 can perceive ROS levels through cysteine-rich regions [133–135]. In the steady state, Nrf2 in the cytoplasm can be degraded by Keap1, and Nrf2 increases rapidly under stress and transfers to the nucleus for transcriptional activity [136]. Mitoquinone (MitoQ) is a mitochondrial-targeted antioxidant and can cause a sharp decline in Keap1 in cells, prompting more Nrf2 to be transmitted to the nucleus to produce an antioxidant response. The effect was confirmed in subarachnoid hemorrhage (SAH) animal model experiments [137]. Nrf2 can also play a protective role as a therapeutic target in astrocytes. There are seven functional domains of Nrf2 (neh1-neh7) that regulate its transcriptional activity and stability [138]. Kelch-like ECH-associated protein 1 (Keap1) is an inhibitor of Nrf2 [139, 140] and interacts with Nrf2 through neh2 domain [141]. Early studies believed that Keap1 inhibition was the main mechanism to activate astrocytes. Recent studies have found that mild oxidative stress (nonlethal oxidative stress) can also activate Nrf2 independently through neh5 transactivation domain [142]. In addition to the various regulatory factors mentioned above, there are other Keap1/Nrf2 pathway regulators such as microRNA-592 (miR-592) [143], eriodictyol [144], and tripartite motif 16 (TRIM16) [145]. These regulatory factors can act on Keap1/Nrf2/ARE pathway to play the role of antioxidant stress, so as to treat or alleviate neurological disorders (Figure 2).

The article "Targeting Molecular Mediators of Ferroptosis and Oxidative Stress for Neurological Disorders" was published in 2022. Journal: Oxid Med Cell Longev.

### 4.2. NADPH- and NOX-Mediated Oxidative Stress

Nicotinamide adenine dinucleotide-phosphate (NADPH) is a coenzyme, which is the product of the final electron acceptor NADP + after receiving electrons. It participates in a variety of biochemical reactions as a hydrogen transmitter in vivo. Studies have confirmed that NADPH can resist oxidative stress and improve energy metabolism, so as to play a neuroprotective role in stroke [146]. NADPH oxidases (NOXs) have 7 kinds of subtypes.

H_2_O_2_ can interact with mutant huntingtin in the brain of HD patients [147]. The activity of NOX can be measured by lucigenin-enhanced luminescence method [148]. The heterozygous huntingtin (HTT) and Cd can induce cytotoxicity which will cause NOXs-mediated oxidative stress. As an exogenous antioxidant and NOX inhibitor, apocynin can block the process of oxidative stress in the process of HD [149]. So far, there are still few studies on the role of NOX in the process of HD. As a potential therapeutic target of HD, the mechanism of NOX and its way of alleviating HD patients deserve further exploration.

Studies found that the cerebellum is an important participant in mental illness and is affected by oxidative stress. Schiavone et al. found that inhibition of NOX during brain maturation can prevent the development of psychotic behavioral dysfunction. Administration of ketamine to the postpartum mouse model can enhance oxidative stress and reduce IL-10 in this region [150]. In recent years, many compounds that inhibit NOX have been studied for the treatment of neurological disorders, and Ganguly et al. [191] reviewed the relationship between NOX and AD, and summarized drug trials of NOX inhibitors in Alzheimer's disease and its precursor conditions. The results displayed that the activity of NOX increased in the brain of mouse models with neurodegenerative diseases and AD patients [192-194]. However, the effects of NOX inhibitors and their precursors are not satisfactory, and the therapeutic results of these naturally obtained compounds for AD are quite variable, including berberine and blueberry-derived polyphenols. Because of the complexity of neurological disorders, the study of NOX inhibitors can provide a new direction for the treatment of neurological disorders (Figure 2).

The article "Targeting Molecular Mediators of Ferroptosis and Oxidative Stress for Neurological Disorders" was published in 2022. Journal: Oxid Med Cell Longev.

### 4.3. Other Mediators and Potential Therapeutic Agents

In this part, we mainly summarize three common regulators of targeted oxidative stress in neurological disorders. In addition to the above three common regulators, other regulators can be used to treat or relieve the symptoms of neurological disorders, such as PINK1, Ca^2+^, Sigma-1 receptor (sig-1R), peroxidase (prx), toll-like receptors (TLRs), and alarmins/c-jun N-terminal kinase (JNK) [151]. PINK1 is a mitochondrial-targeted E3 ubiquitin ligase, whose deficiency can lead to mitochondrial damage, oxidative stress, and exert neuroprotective effects by activating Parkin. Ca^2+^ can consume GSH to regulate cell death [152]. Sigma-1 receptor (sig-1R) [153, 154] is a mitochondrial endoplasmic reticulum chaperon that can regulate cell pathophysiological processes. Peroxidase (prx) can scavenge H_2_O_2_ to regulate redox signal transduction and play a protective role [155]. In addition, Toll-like receptors (TLRs) are also closely related to the injury of a variety of neurological disorders and can promote microglia to release neuroprotective agents through conduction [156]. Anfinogenova et al. [157] described the role of alarmins/c-jun N-terminal kinase (JNK) signaling transduction in cerebrovascular inflammation and summarized the therapeutic strategies of intracellular anti-JNK, which provided ideas for the strategies of JNK in the treatment of neurological disorders.

As an important regulator of oxidative stress, N-acetylcysteine (NAC) is a synthetic derivative of the endogenous amino acid L-cysteine and a precursor of GSH. GSH is a key factor in the clearance of ROS. Studies have shown that NAC mainly relies on GSH to exert its indirect antioxidant capacity, but this capacity is weak [158–160]. The direct antioxidant capacity of NAC depends on its nucleophilic free sulfhydryl group [158]. A large amount of preclinical evidence shows that NAC can play a therapeutic role in CNS by regulating glutamate homeostasis [161]. Glutamate is the main excitatory neurotransmitter in the nervous system. Its overexcitation will lead to neuronal damage [162]. Extracellular glutamate is regulated by glutamate transporter-1 (GLT1), glutamate aspartate transporter (GLAST), and the systemXc^−^ to maintain homeostasis. Experiments have confirmed that NAC can activate systemXc^−^ [163, 164] and induce the expression of GLT1 [165].

The article "Targeting Molecular Mediators of Ferroptosis and Oxidative Stress for Neurological Disorders" was published in 2022. Journal: Oxid Med Cell Longev.

As a precursor of GSH, NAC plays a beneficial role in the pathology and sequelae of TBI. Previous studies have shown that the administration time of NAC affects the therapeutic effect of NAC on TBI. Previous studies have shown that the administration time of NAC affects the therapeutic effect of NAC on TBI. In the 3-day TBI model, NAC administration 15-60 minutes after the injury can reduce the inflammatory response [166, 167], and NAC administration 12 hours after controlled cortical impact (CCI)-induced injury can reduce the level of ROS by increasing GSH [168], and oral NAC treatment within 24 hours after injury can alleviate the sequelae of TBI, such as confusion, headache, and abnormal sleep [169]. Recent studies have also found that the use of antioxidant dual therapy targeting antioxidant stress has a significant effect on the symptoms of TBI and improves the functional outcome [170]. For example, the use of NAC and sulforaphane (SFN) dual therapy can reduce TNF, IL, and other neuroinflammatory markers. In addition, the dual therapy of NAC + SPF has also been proved to be effective in alleviating epilepsy after SE [171]. In recent studies, c57bl/6 (wild type, WT) mice and CCL5 knockout (CCL5-KO) mice were used to induce mild brain injury and establish a weight drop model [172], which is a novel TBI model that can simulate the full spectrum of human TBI, mainly focusing on simulating diffuse brain injury. In the weight drop model, NAC can significantly alleviate the symptoms of decreased memory and learning ability after trauma and increase the level of Gpx1 in the hippocampus of mice [173]. With the application of nanomaterials in biomedicine, it is found that embedding NAC eluted poly (d,l-lactide-co-glycolide) (PLGA) nanofibers into scaffolds can effectively improve the shelf life of drugs and reduce systemic side effects. At the same time, it can give full play to the neuroprotective effect of NAC and the cell proliferation of nanosystems [174], which provides a broad prospect for the application of nanosystems in nerve repair. For example, neutral hydroxyl-terminated polyamide (PAMAM) dendrimers have shown great potential as nanocarriers in multiple brain injury models [175].

The article "Targeting Molecular Mediators of Ferroptosis and Oxidative Stress for Neurological Disorders" was published in 2022. Journal: Oxid Med Cell Longev.

## 5. Conclusion

In this review, we summarize the relevant mechanisms of ferroptosis and some regulators of targeted oxidative stress in the treatment of neurological disorders. In the process of searching the literature, we find that oxidative stress and neurological disorders are closely related to the role of mitochondria (Figure 2), but the connection is very complex and lacks a systematic and clear mechanism. Ferroptosis may be a key mechanism to study the connection (Figure 1). For future research on neurological disorders, the role of mitochondria and the mechanism of ferroptosis will be the focus and hotspot of research. In addition, in view of the harmfulness of neurological disorders and the complexity of oxidative stress and ferroptosis, future research on the molecular mediators targeting oxidative stress and ferroptosis should pay more attention to the underlying mechanisms, so as to provide a theoretical basis for the treatment of neurological disorders.

## Figures and Tables

**Figure 1:** A schematic summary of ferroptosis mechanisms in neurological disorders. Lipid peroxidation and iron homeostasis are currently recognized as important mechanisms affecting ferroptosis. In cells, under the action of ACSL4, PRO, and ALOX, PUFA generates PLOOH through a series of biochemical reactions, which then generates PLOO, leading to lipid peroxidation and eventually ferroptosis. GPX4 can reduce PLOOH to PLOH to inhibit lipid peroxidation. In addition, GPX4 is regulated by the cofactor GSH. When GSH is exhausted, GPX4 will be inactivated. Glutamate and cystine generate GSH through systemX_C_^−^ and GSH can be oxidized to GSSG. Mitochondria generate ROS through ETC in TCA cycle, which leads to oxidative stress and eventually ferroptosis. Fe^2+^ is oxidized to Fe^3+^ after being absorbed in the duodenum. Fe^3+^ enters the cell by combining with Tf and Tfr to form a complex. Iron ions decomposed from the endosome can leave the cell through FPN protein on the cell membrane, and other iron ions enter the unstable iron pool. Tf-Tfr complex leaves the cell for the next cycle. Under pathological conditions (neurological disorders), excessive Fe^2+^ will participate in Fenton reaction to produce a large amount of ROS, which will lead to ferroptosis. Abbreviations: AA: arachidonic acid; AdA: adrenic acid; ACLS4: acyl-CoA synthetase long chain family member 4; ALOXs: lipoxygenases; CoA: coenzyme A; DPI7: diphenyleneiodonium chloride7; ETC: electron transport chain; FPn: ferroportin; GPX4: glutathione peroxidase 4; GSH: glutathione; GSSG: oxidized glutathione; LPCAT3: lysophosphatidylcholine acyltransferase 3; OGDH: oxoglutarate dehydrogenase; PL: phospholipid; POR: cytochrome p450 oxidoreductase; PLOOH: phospholipid hydroperoxides; PUFA: polyunsaturated fatty acids; RSL3: (1S,3R)-RSL3; ROS: reactive oxygen species; STEAP3: STEAP family member 3; Tf: transferrin; Tfr: transferrin receptor; TZD: thiazolidinediones; TCA: tricarboxylic acid.

The article "Targeting Molecular Mediators of Ferroptosis and Oxidative Stress for Neurological Disorders" was published in 2022. Journal: Oxid Med Cell Longev.

**Figure 2:** The top schematic is a summary of oxidative stress mechanisms in neurological disorders. Under homeostatic conditions, Nrf2 binds with Keap1 and remains inactive. Nrf2-keap1 is also regulated by PI3K-Akt pathway. Under pathological conditions (neurological disorders) cause oxidative stress, Nrf2 and Keap1 will be separated. Nrf2 enters the nucleus and combines with MAF and ARE to activate antioxidant metabolic genes and play an antioxidant role. In addition, Nrf2 can activate GPX4 and be inhibited by Keap1. Both TCA cycle in mitochondria and Fenton reaction involving Fe^2+^ can cause oxidative stress by producing ROS. NAC, as a precursor of GPX4 and L-cysteine, affects oxidative stress through systemX_C_^−^ and GPX4. In addition, NAC can interfere with glutamate homeostasis and participate in the occurrence of a variety of nervous system diseases. NOX can produce ROS and cause oxidative stress under the action of a variety of regulatory factors. The bottom table is a summary of several molecules that affect oxidative stress in neurological disorders, including their action targets, action modes, and action results. Abbreviations: Akt: protein kinase B; ARE: antioxidant response element; ETC: electron transport chain; GPX4: glutathione peroxidase 4; Keap1: Kelch-like ECH-associated protein 1; Maf: musculoaponeurotic fibrosarcoma oncogene homolog; NAC: N-acetylcysteine; NOX: nicotinamide adenine dinucleotide phosphate oxidases; NADP: nicotinamide adenine dinucleotide phosphate; Nrf2: NF-E2-related factor 2; PI3K: phosphatidylinositol-3-kinase; ROS: reactive oxygen species; TCA: tricarboxylic acid.

**Table 1:** Ferroptosis-induced effects or altered physiology in neurological disorders.

Object	Effect/physiological changes	Reference
Alzheimer's disease (AD) model	Induce neuronal death and memory impairment	[80]
Rat corticostriatal brain slices	Induce the oxidative destruction of PUFA	[94]
Cuprizone model	Induce oligodendrocyte loss and demyelination	[176]
In vivo TBI model/mice model with TBI	Induce inflammation and neuronal death	[177]
Transient cerebral ischemia model	Induce neuronal death	[178]
Type 1 diabetes rat model	Induce cognitive dysfunctions	[179]
Lund human mesencephalic cells/mice model with PD	Induce dopaminergic cell death	[180]
Mitochondrion	Shrinkage of mitochondria with enhanced mitochondrial membrane density, mitochondrial volume reduction, vanishing of mitochondria crista, outer mitochondrial membrane rupture	[181]

The article "Targeting Molecular Mediators of Ferroptosis and Oxidative Stress for Neurological Disorders" was published in 2022. Journal: Oxid Med Cell Longev.

## References

[1] Dixon S. J. S. J., Lemberg K. M., Lamprecht M. R. (2012). Ferroptosis: An Iron-Dependent Form of Nonapoptotic Cell Death. *Cell*.

[2] Chen X., Li J., Kang R., Klionsky D. J., Tang D. (2021). Ferroptosis: machinery and regulation. *Autophagy*.

[3] Yu Y., Yan Y., Niu F. (2021). Ferroptosis: a cell death connecting oxidative stress, inflammation and cardiovascular diseases. *Cell Death Discovery*.

[4] Xu S., He Y., Lin L., Chen P., Chen M., Zhang S. (2021). The emerging role of ferroptosis in intestinal disease. *Cell Death & Disease*.

[5] Li J., Cao F., Yin H. L. (2020). Ferroptosis: past, present and future. *Cell Death & Disease*.

[6] Ren J., Li C., Yan X. L., Qu Y., Yang Y., Guo Z. N. (2021). Crosstalk between oxidative stress and ferroptosis/oxytosis in ischemic stroke: possible targets and molecular mechanisms. *Oxidative Medicine and Cellular Longevity*.

[7] Feigin V. L., Vos T., Nichols E. (2020). The global burden of neurological disorders: translating evidence into policy. *The Lancet Neurology*.

[8] Winkler A. S. (2020). The growing burden of neurological disorders in low-income and middle-income countries: priorities for policy making. *Lancet Neurology*.

[9] Schmitt A., Xu W., Bucher P. (2021). Dimethyl fumarate induces ferroptosis and impairs NF-*κ*B/STAT3 signaling in DLBCL. *Blood*.

[10] Li Y., Wang X., Huang Z. (2021). CISD3 inhibition drives cystine-deprivation induced ferroptosis. *Cell Death & Disease*.

[11] Lei G., Zhuang L., Gan B. (2021). mTORC1 and ferroptosis: regulatory mechanisms and therapeutic potential. *BioEssays*.

[12] Koppula P., Zhuang L., Gan B. (2021). Cystine transporter SLC7A11/xCT in cancer: ferroptosis, nutrient dependency, and cancer therapy. *Protein & Cell*.

[13] Qu W., Cheng Y., Peng W. (2022). Targeting iNOS alleviates early brain injury after experimental subarachnoid hemorrhage via promoting ferroptosis of M1 microglia and reducing neuroinflammation. *Molecular Neurobiology*.

[14] Zhao Y., Li Y., Zhang R., Wang F., Wang T., Jiao Y. (2020). The role of erastin in ferroptosis and its prospects in cancer therapy. *OncoTargets and therapy*.

[15] Zhang H., Jiao W., Cui H., Sun Q., Fan H. (2021). Combined exposure of alumina nanoparticles and chronic stress exacerbates hippocampal neuronal ferroptosis via activating IFN-*γ*/ASK1/JNK signaling pathway in rats. *Journal of Hazardous Materials*.

The article "Targeting Molecular Mediators of Ferroptosis and Oxidative Stress for Neurological Disorders" was published in 2022. Journal: Oxid Med Cell Longev.

[16] Wang Y., Zhao Y., Ye T., Yang L., Shen Y., Li H. (2021). Ferroptosis signaling and regulators in atherosclerosis. *Frontiers in cell and developmental biology*.

[17] Liu J., Kang R., Tang D. (2021). Signaling pathways and defense mechanisms of ferroptosis. *The FEBS Journal*.

[18] Xu S., Wu B., Zhong B. (2021). Naringenin alleviates myocardial ischemia/reperfusion injury by regulating the nuclear factor-erythroid factor 2-related factor 2 (Nrf2) /system xc-/ glutathione peroxidase 4 (GPX4) axis to inhibit ferroptosis. *Bioengineered*.

[19] Forman H. J., Zhang H. (2021). Targeting oxidative stress in disease: promise and limitations of antioxidant therapy. *Nature Reviews. Drug Discovery*.

[20] Singh A., Kukreti R., Saso L., Kukreti S. (2019). Oxidative stress: a key modulator in neurodegenerative diseases. *Molecules*.

[21] Wang L., Liu Y., du T. (2020). ATF3 promotes erastin-induced ferroptosis by suppressing system Xc^−^. *Cell Death and Differentiation*.

[22] Maiorino M., Conrad M., Ursini F. (2018). GPx4, lipid peroxidation, and cell death: discoveries, rediscoveries, and open issues. *Antioxidants & Redox Signaling*.

[23] Yang S., Lian G. (2020). ROS and diseases: role in metabolism and energy supply. *Molecular and Cellular Biochemistry*.

[24] Tripathi R., Gupta R., Sahu M. (2021). Free radical biology in neurological manifestations: mechanisms to therapeutics interventions. *Environmental Science and Pollution Research International*.

[25] Ni S., Yuan Y., Kuang Y., Li X. (2022). Iron metabolism and immune regulation. *Frontiers in Immunology*.

[26] Wang S., Luo J., Zhang Z. (2018). Iron and magnetic: new research direction of the ferroptosis-based cancer therapy. *American Journal of Cancer Research*.

[27] Geng Z., Guo Z., Guo R., Ye R., Zhu W., Yan B. (2021). Ferroptosis and traumatic brain injury. *Brain Research Bulletin*.

[28] Haschka D., Hoffmann A., Weiss G. (2021). Iron in immune cell function and host defense. *Seminars in Cell & Developmental Biology*.

[29] Tsuneda T. (2020). Fenton reaction mechanism generating no OH radicals in Nafion membrane decomposition. *Scientific Reports*.

[30] Fenton H. J. H. (1894). LXXIII.—Oxidation of tartaric acid in presence of iron. *Journal of the Chemical Society*.

[31] Wang H., Liu C., Zhao Y., Gao G. (2020). Mitochondria regulation in ferroptosis. *European Journal of Cell Biology*.

[32] Friedman J. R., Nunnari J. (2014). Mitochondrial form and function. *Nature*.

[33] Connolly B. S., Lang A. E. (2014). Pharmacological treatment of Parkinson Disease. *JAMA*.

[34] Moreau C., Duce J. A., Rascol O. (2018). Iron as a therapeutic target for Parkinson’s disease. *Movement Disorders*.

The article "Targeting Molecular Mediators of Ferroptosis and Oxidative Stress for Neurological Disorders" was published in 2022. Journal: Oxid Med Cell Longev.

[35] Chipuk J. E., Mohammed J. N., Gelles J. D., Chen Y. (2021). Mechanistic connections between mitochondrial biology and regulated cell death. *Developmental Cell*.

[36] Xu C., Sun S., Johnson T. (2021). The glutathione peroxidase Gpx4 prevents lipid peroxidation and ferroptosis to sustain Treg cell activation and suppression of antitumor immunity. *Cell Reports*.

[37] Yang M., Tsui M. G., Tsang J. K. W. (2022). Involvement of FSP1-CoQ_10_-NADH and GSH-GPx-4 pathways in retinal pigment epithelium ferroptosis. *Cell Death & Disease*.

[38] Doll S., Freitas F. P., Shah R. (2019). FSP1 is a glutathione-independent ferroptosis suppressor. *Nature (London)*.

[39] Sun X., Ou Z., Chen R. (2016). Activation of the p62-Keap1-NRF2 pathway protects against ferroptosis in hepatocellular carcinoma cells. *Hepatology*.

[40] Tan Q., Fang Y., Gu Q. (2021). Mechanisms of modulation of ferroptosis and its role in central nervous system diseases. *Frontiers in Pharmacology*.

[41] Rui T., Wang H., Li Q. (2021). Deletion of ferritin H in neurons counteracts the protective effect of melatonin against traumatic brain injury-induced ferroptosis. *Journal of Pineal Research*.

[42] Cai Y., Yang Z. (2021). Ferroptosis and its role in epilepsy. *Frontiers in Cellular Neuroscience*.

[43] Lane D., Metselaar B., Greenough M., Bush A. I., Ayton S. J. (2021). Ferroptosis and NRF2: an emerging battlefield in the neurodegeneration of Alzheimer’s disease. *Essays in Biochemistry*.

[44] Fearnley J. M., Lees A. J. (1991). Ageing and Parkinson’s disease: substantia nigra regional selectivity. *Brain*.

[45] Rinne J. O., Rummukainen J., Paljärvi L., Säkö E., Mölsä P., Rinne U. K. (1989). Neuronal loss in the substantia nigra in patients with Alzheimer’s disease and Parkinson’s disease in relation to extrapyramidal symptoms and dementia. *Progress in Clinical and Biological Research*.

[46] Antony P. M., Diederich N. J., Krüger R., Balling R. (2013). The hallmarks of Parkinson’s disease. *The FEBS Journal*.

[47] Ward R. J. P., Zucca F. A., Duyn J. H., Crichton R. R., Zecca L. (2014). The role of iron in brain ageing and neurodegenerative disorders. *Lancet Neurology*.

[48] Sian J., Dexter D. T., Lees A. J. (1994). Alterations in glutathione levels in Parkinson’s disease and other neurodegenerative disorders affecting basal ganglia. *Annals of Neurology*.

[49] Cassarino D. S., Fall C. P., Swerdlow R. H. (1997). Elevated reactive oxygen species and antioxidant enzyme activities in animal and cellular models of Parkinson's disease. *Biochimica et Biophysica Acta*.

[50] Dexter D., Carter C., Agid F. (1986). LIPID PEROXIDATION AS CAUSE OF NIGRAL CELL DEATH IN PARKINSON'S DISEASE. *The Lancet*.

The article "Targeting Molecular Mediators of Ferroptosis and Oxidative Stress for Neurological Disorders" was published in 2022. Journal: Oxid Med Cell Longev.

[51] Tian Y., Lu J., Hao X. (2020). FTH1 inhibits ferroptosis through ferritinophagy in the 6-OHDA model of Parkinson’s disease. *Neurotherapeutics*.

[52] Guiney S. J., Adlard P. A., Bush A. I., Finkelstein D. I., Ayton S. (2017). Ferroptosis and cell death mechanisms in Parkinson's disease. *Neurochemistry International*.

[53] Weiland A., Wang Y., Wu W. (2019). Ferroptosis and its role in diverse brain diseases. *Molecular Neurobiology*.

[54] Zhang P., Chen L., Zhao Q. (2020). Ferroptosis was more initial in cell death caused by iron overload and its underlying mechanism in Parkinson’s disease. *Free Radical Biology & Medicine*.

[55] Ganguly U., Banerjee A., Chakrabarti S. S. (2020). Interaction of *α*-synuclein and Parkin in iron toxicity on SH-SY5Y cells: implications in the pathogenesis of Parkinson’s disease. *Biochemical Journal*.

[56] Stefanis L. (2012). Synuclein in Parkinson's Disease. *Cold Spring Harb Perspect Med*.

[57] Angelova P. R., Choi M. L., Berezhnov A. V. (2020). Alpha synuclein aggregation drives ferroptosis: an interplay of iron, calcium and lipid peroxidation. *Cell Death and Differentiation*.

[58] Miotto G., Rossetto M., di Paolo M. L. (2020). Insight into the mechanism of ferroptosis inhibition by ferrostatin-1. *Redox Biology*.

[59] DeTure M. A., Dickson D. W. (2019). The neuropathological diagnosis of Alzheimer’s disease. *Molecular Neurodegeneration*.

[60] Mills E., Dong X. P., Wang F., Xu H. (2010). Mechanisms of brain iron transport: insight into neurodegeneration and CNS disorders. *Future Medicinal Chemistry*.

[61] Masaldan S., Bush A. I., Devos D., Rolland A. S., Moreau C. (2019). Striking while the iron is hot: Iron metabolism and ferroptosis in neurodegeneration. *Free Radical Biology and Medicine*.

[62] Duce J. A., Tsatsanis A., Cater M. A. (2010). Iron-export ferroxidase activity of *β*-amyloid precursor protein is inhibited by zinc in Alzheimer’s disease. *Cell*.

[63] Jellinger K., Paulus W., Grundke-Iqbal I., Riederer P., Youdim M. B. H. (1990). Brain iron and ferritin in Parkinson’s and Alzheimer’s diseases. *Journal of Neural Transmission. Parkinson's Disease and Dementia Section*.

[64] Smith M. A., Harris P. L. R., Sayre L. M., Perry G. (1997). Iron accumulation in Alzheimer disease is a source of redox-generated free radicals. *Proceedings of the National Academy of Sciences of the United States of America*.

[65] Ayton S., Lei P., Hare D. J. (2015). Parkinson's disease iron deposition caused by nitric oxide-induced loss of -Amyloid Precursor Protein. *The Journal of Neuroscience*.

[66] Connor J. R., Snyder B. S., Beard J. L., Fine R. E., Mufson E. J. (1992). Regional distribution of iron and iron-regulatory proteins in the brain in aging and Alzheimer’s disease. *Journal of Neuroscience Research*.

The article "Targeting Molecular Mediators of Ferroptosis and Oxidative Stress for Neurological Disorders" was published in 2022. Journal: Oxid Med Cell Longev.

[67] Good P. F., Perl D. P., Bierer L. M., Schmeidler J. (1992). Selective accumulation of aluminum and iron in the neurofibrillary tangles of Alzheimer’s disease: a laser microprobe (LAMMA) study. *Annals of Neurology*.

[68] Ayton S., Wang Y., Diouf I. (2020). Brain iron is associated with accelerated cognitive decline in people with Alzheimer pathology. *Molecular Psychiatry*.

[69] Stockwell B. R., Friedmann Angeli J. P., Bayir H. (2017). Ferroptosis: a regulated cell death nexus linking metabolism, redox biology, and disease. *Cell*.

[70] Williams T. I., Lynn B. C., Markesbery W. R., Lovell M. A. (2006). Increased levels of 4-hydroxynonenal and acrolein, neurotoxic markers of lipid peroxidation, in the brain in Mild Cognitive Impairment and early Alzheimer's disease. *Neurobiology of Aging*.

[71] Butterfield D. A., Poon H. F., St. Clair D. (2006). Redox proteomics identification of oxidatively modified hippocampal proteins in mild cognitive impairment: insights into the development of Alzheimer’s disease. *Neurobiology of Disease*.

[72] Derry P. J., Hegde M. L., Jackson G. R. (2020). Revisiting the intersection of amyloid, pathologically modified tau and iron in Alzheimer's disease from a ferroptosis perspective. *Progress in Neurobiology*.

[73] Mandal P. K., Saharan S., Tripathi M., Murari G. (2015). Brain Glutathione Levels - A Novel Biomarker for Mild Cognitive Impairment and Alzheimer's Disease. *Biological Psychiatry*.

[74] Ashraf A., Jeandriens J., Parkes H. G., So P. W. (2020). Iron dyshomeostasis, lipid peroxidation and perturbed expression of cystine/glutamate antiporter in Alzheimer's disease: Evidence of ferroptosis. *Redox Biology*.

[75] Habib E., Linher-Melville K., Lin H. X., Singh G. (2015). Expression of xCT and activity of system x_c_^−^ are regulated by NRF2 in human breast cancer cells in response to oxidative stress. *Redox Biology*.

[76] Correa F., Ljunggren E., Mallard C., Nilsson M., Weber S. G., Sandberg M. (2011). The Nrf2-inducible antioxidant defense in astrocytes can be both up- and down-regulated by activated microglia: involvement of p38 MAPK. *Glia*.

[77] Hambright W. S., Fonseca R. S., Chen L., Na R., Ran Q. (2017). Ablation of ferroptosis regulator glutathione peroxidase 4 in forebrain neurons promotes cognitive impairment and neurodegeneration. *Redox Biology*.

[78] Stankowski J. N., Dawson V. L., Dawson T. M. (2012). Ironing out tau's role in parkinsonism. *Nature Medicine*.

[79] Lei P., Ayton S., Finkelstein D. I. (2012). Tau deficiency induces parkinsonism with dementia by impairing APP-mediated iron export. *Nature Medicine*.

The article "Targeting Molecular Mediators of Ferroptosis and Oxidative Stress for Neurological Disorders" was published in 2022. Journal: Oxid Med Cell Longev.

[80] Bao W. D., Pang P., Zhou X. T. (2021). Loss of ferroportin induces memory impairment by promoting ferroptosis in Alzheimer's disease. *Cell Death and Differentiation*.

[81] Park M. W., Cha H. W., Kim J. (2021). NOX4 promotes ferroptosis of astrocytes by oxidative stress-induced lipid peroxidation via the impairment of mitochondrial metabolism in Alzheimer's diseases. *Redox Biology*.

[82] Bhatia R., Chakrabarti S. S., Kaur U., Parashar G., Banerjee A., Rawal R. K. (2021). Multi-target directed ligands (MTDLs): promising coumarin hybrids for Alzheimer’s disease. *Current Alzheimer Research*.

[83] Ashraf A., So P. W. (2020). Spotlight on ferroptosis: iron-dependent cell death in Alzheimer’s disease. *Frontiers in Aging Neuroscience*.

[84] Ross C. A., Tabrizi S. J. (2011). Huntington’s disease: from molecular pathogenesis to clinical treatment. *Lancet Neurology*.

[85] Mi Y., Gao X., Xu H., Cui Y., Zhang Y., Gou X. (2019). The emerging roles of ferroptosis in Huntington’s disease. *Neuromolecular Medicine*.

[86] Pigeon C., Ilyin G., Courselaud B. (2001). A New Mouse Liver-specific Gene, Encoding a Protein Homologous to Human Antimicrobial Peptide Hepcidin, Is Overexpressed during Iron Overload. *The Journal of Biological Chemistry*.

[87] Zhang H., Ostrowski R., Jiang D. (2021). Hepcidin promoted ferroptosis through iron metabolism which is associated with DMT1 signaling activation in early brain injury following subarachnoid hemorrhage. *Oxidative Medicine and Cellular Longevity*.

[88] Geng N., Shi B. J., Li S. L. (2018). Knockdown of ferroportin accelerates erastin-induced ferroptosis in neuroblastoma cells. *European Review for Medical and Pharmacological Sciences*.

[89] Qian Z. M., Ke Y. (2020). Hepcidin and its therapeutic potential in neurodegenerative disorders. *Medicinal Research Reviews*.

[90] Chen J., Marks E., Lai B. (2013). Iron accumulates in Huntington’s disease neurons: protection by deferoxamine. *PLoS One*.

[91] Paul B. D., Sbodio J. I., Xu R. (2014). Cystathionine *γ*-lyase deficiency mediates neurodegeneration in Huntington's disease. *Nature*.

[92] Klepac N., Relja M., Klepac R., Hećimović S., Babić T., Trkulja V. (2007). Oxidative stress parameters in plasma of Huntington’s disease patients, asymptomatic Huntington’s disease gene carriers and healthy subjects : a cross-sectional study. *Journal of Neurology*.

[93] Cardoso B. R., Hare D. J., Bush A. I., Roberts B. R. (2017). Glutathione peroxidase 4: a new player in neurodegeneration?. *Molecular Psychiatry*.

[94] Skouta R., Dixon S. J., Wang J. (2014). Ferrostatins inhibit oxidative lipid damage and cell death in diverse disease models. *Journal of the American Chemical Society*.

The article "Targeting Molecular Mediators of Ferroptosis and Oxidative Stress for Neurological Disorders" was published in 2022. Journal: Oxid Med Cell Longev.

[95] Jiao H., Yang H., Yan Z. (2021). Traditional Chinese formula Xiaoyaosan alleviates depressive-like behavior in CUMS mice by regulating PEBP1-GPX4-mediated ferroptosis in the hippocampus. *Neuropsychiatric Disease and Treatment*.

[96] Chen W. L., Xie B., Zhang C. (2013). Antidepressant-like and anxiolytic-like effects of hydrogen sulfide in behavioral models of depression and anxiety. *Behavioural Pharmacology*.

[97] Wang Y., Wang S., Xin Y. (2021). Hydrogen sulfide alleviates the anxiety-like and depressive-like behaviors of type 1 diabetic mice via inhibiting inflammation and ferroptosis. *Life Sciences*.

[98] Black C. N., Bot M., Scheffer P. G., Cuijpers P., Penninx B. W. J. H. (2015). Is depression associated with increased oxidative stress? A systematic review and meta-analysis. *Psychoneuroendocrinology*.

[99] Bhatt S., Nagappa A. N., Patil C. R. (2020). Role of oxidative stress in depression. *Drug Discovery Today*.

[100] Sriram C. S., Jangra A., Gurjar S. S., Mohan P., Bezbaruah B. K. (2016). Edaravone abrogates LPS-induced behavioral anomalies, neuroinflammation and PARP-1. *Physiology & Behavior*.

[101] Dang R., Wang M., Li X. (2022). Edaravone ameliorates depressive and anxiety-like behaviors via Sirt1/Nrf2/HO-1/Gpx4 pathway. *Journal of Neuroinflammation*.

[102] Benjamin E. J., Muntner P., Alonso A. (2019). Heart disease and stroke statistics-2019 update: a report from the American Heart Association. *Circulation*.

[103] Zhang Y., Lu X., Tai B., Li W., Li T. (2021). Ferroptosis and its multifaceted roles in cerebral stroke. *Frontiers in Cellular Neuroscience*.

[104] Jin Y., Zhuang Y., Liu M., Che J., Dong X. (2021). Inhibiting ferroptosis: a novel approach for stroke therapeutics. *Drug Discovery Today*.

[105] Chen G., Li L., Tao H. (2021). Bioinformatics identification of ferroptosis-related biomarkers and therapeutic compounds in ischemic stroke. *Frontiers in Neurology*.

[106] Karuppagounder S. S., Alin L., Chen Y. (2018). N-acetylcysteine targets 5 lipoxygenase-derived, toxic lipids and can synergize with prostaglandin E2 to inhibit ferroptosis and improve outcomes following hemorrhagic stroke in mice. *Annals of Neurology*.

[107] Olmez I., Ozyurt H. (2012). Reactive oxygen species and ischemic cerebrovascular disease. *Neurochemistry International*.

[108] Guan X., Li X., Yang X. (2019). The neuroprotective effects of carvacrol on ischemia/reperfusion-induced hippocampal neuronal impairment by ferroptosis mitigation. *Life Sciences*.

[109] Cui Y., Zhang Y., Zhao X. (2021). ACSL4 exacerbates ischemic stroke by promoting ferroptosis-induced brain injury and neuroinflammation. *Brain, Behavior, and Immunity*.

The article "Targeting Molecular Mediators of Ferroptosis and Oxidative Stress for Neurological Disorders" was published in 2022. Journal: Oxid Med Cell Longev.

[110] An S. J., Kim T. J., Yoon B. W. (2017). Epidemiology, risk factors, and clinical features of intracerebral hemorrhage: an update. *Journal of Stroke*.

[111] Xiong X. Y., Wang J., Qian Z. M., Yang Q. W. (2014). Iron and intracerebral hemorrhage: from mechanism to translation. *Translational Stroke Research*.

[112] Okauchi M., Hua Y., Keep R. F., Morgenstern L. B., Schallert T., Xi G. (2010). Deferoxamine treatment for intracerebral hemorrhage in aged rats: therapeutic time window and optimal duration. *Stroke*.

[113] Zille M., Karuppagounder S. S., Chen Y. (2017). Neuronal death after hemorrhagic stroke in vitro and in vivo shares features of ferroptosis and necroptosis. *Stroke*.

[114] Alim I., Caulfield J. T., Chen Y. (2019). Selenium drives a transcriptional adaptive program to block ferroptosis and treat stroke. *Cell*.

[115] Hu X., Xu Y., Xu H. (2021). Progress in understanding ferroptosis and its targeting for therapeutic benefits in traumatic brain and spinal cord injuries. *Frontiers in Cell and Developmental Biology*.

[116] Vos P. E., Diaz-Arrastia R. (2015). *Traumatic brain injury*.

[117] Tyurin V. A., Tyurina Y. Y., Borisenko G. G. (2000). Oxidative stress following traumatic brain injury in rats: quantitation of biomarkers and detection of free radical intermediates. *Journal of Neurochemistry*.

[118] Bayir H., Kagan V. E., Tyurina Y. Y. (2002). Assessment of antioxidant reserves and oxidative stress in cerebrospinal fluid after severe traumatic brain injury in infants and children. *Pediatric Research*.

[119] Xie B. S., Wang Y. Q., Lin Y. (2019). Inhibition of ferroptosis attenuates tissue damage and improves long-term outcomes after traumatic brain injury in mice. *CNS Neuroscience & Therapeutics*.

[120] Wanet A., Tacheny A., Arnould T., Renard P. (2012). miR-212/132 expression and functions: within and beyond the neuronal compartment. *Nucleic Acids Research*.

[121] Quiles Del Rey M., Mancias J. D. (2019). NCOA4-mediated ferritinophagy: a potential link to neurodegeneration. *Frontiers in Neuroscience*.

[122] Sun S., Han X., Li X. (2018). MicroRNA-212-5p prevents dopaminergic neuron death by inhibiting SIRT2 in MPTP-induced mouse model of Parkinson’s disease. *Frontiers in Molecular Neuroscience*.

[123] Xiao X., Jiang Y., Liang W. (2019). miR-212-5p attenuates ferroptotic neuronal death after traumatic brain injury by targeting Ptgs2. *Molecular Brain*.

[124] Cheng Y., Qu W., Li J. (2022). Ferristatin II, an iron uptake inhibitor, exerts neuroprotection against traumatic brain injury via suppressing ferroptosis. *ACS Chemical Neuroscience*.

[125] Hulbert A. J., Pamplona R., Buffenstein R., Buttemer W. A. (2007). Life and death: metabolic rate, membrane composition, and life span of animals. *Physiological Reviews*.

The article "Targeting Molecular Mediators of Ferroptosis and Oxidative Stress for Neurological Disorders" was published in 2022. Journal: Oxid Med Cell Longev.

[126] Jung K., Kwak M. (2010). The Nrf2 system as a potential target for the development of indirect antioxidants. *Molecules*.

[127] Liu L., Locascio L. M., Doré S. (2019). Critical role of Nrf2 in experimental ischemic stroke. *Frontiers in Pharmacology*.

[128] Zhang L., Wang H. (2017). Targeting the NF-E2-related factor 2 pathway: a novel strategy for traumatic brain injury. *Molecular Neurobiology*.

[129] Calkins M. J., Johnson D. A., Townsend J. A. (2009). The Nrf2/ARE pathway as a potential therapeutic target in neurodegenerative disease. *Antioxidants & Redox Signaling*.

[130] Yang F. Y., Guan Q. K., Cui Y. H., Zhao Z. Q., Rao W., Xi Z. (2012). NAD(P)H quinone oxidoreductase 1 (NQO1) genetic C609T polymorphism is associated with the risk of digestive tract cancer: a meta-analysis based on 21 case-control studies. *European Journal of Cancer Prevention*.

[131] Wild A. C., Moinova H. R., Mulcahy R. T. (1999). Regulation of *γ*-glutamylcysteine synthetase subunit gene expression by the transcription factor Nrf2. *Journal of Biological Chemistry*.

[132] Moinova H. R., Mulcahy R. T. (1999). Up-regulation of the human *γ*-glutamylcysteine synthetase regulatory subunit gene involves binding of Nrf-2 to an electrophile responsive element. *Biochemical and Biophysical Research Communications*.

[133] Zhang D. D., Hannink M. (2003). Distinct cysteine residues in Keap1 are required for Keap1-dependent ubiquitination of Nrf2 and for stabilization of Nrf2 by chemopreventive agents and oxidative stress. *Molecular and Cellular Biology*.

[134] McMahon M., Thomas N., Itoh K., Yamamoto M., Hayes J. D. (2004). Redox-regulated Turnover of Nrf2 Is Determined by at Least Two Separate Protein Domains, the Redox-sensitive Neh2 Degron and the Redox-insensitive Neh6 Degron. *Journal of Biological Chemistry*.

[135] Kobayashi M., Li L., Iwamoto N. (2009). The antioxidant defense system Keap1-Nrf2 comprises a multiple sensing mechanism for responding to a wide range of chemical compounds. *Molecular and Cellular Biology*.

[136] Dodson M., Redmann M., Rajasekaran N. S., Darley-Usmar V., Zhang J. (2015). KEAP1–NRF2 signalling and autophagy in protection against oxidative and reductive proteotoxicity. *Biochemical Journal*.

[137] Zhang T., Wu P., Budbazar E. (2019). Mitophagy reduces oxidative stress via Keap1 (Kelch-like epichlorohydrin-associated protein 1)/Nrf2 (nuclear factor-E2-related factor 2)/PHB2 (prohibitin 2) pathway after subarachnoid hemorrhage in rats. *Stroke*.

[138] Cardozo L. F. M. F., Pedruzzi L. M., Stenvinkel P. (2013). Nutritional strategies to modulate inflammation and oxidative stress pathways via activation of the master antioxidant switch Nrf2. *Biochimie*.

The article "Targeting Molecular Mediators of Ferroptosis and Oxidative Stress for Neurological Disorders" was published in 2022. Journal: Oxid Med Cell Longev.

[139] Itoh K., Wakabayashi N., Katoh Y. (1999). Keap1 represses nuclear activation of antioxidant responsive elements by Nrf2 through binding to the amino-terminal Neh2 domain. *Genes & Development*.

[140] Wakabayashi N., Itoh K., Wakabayashi J. (2003). *Keap1* -null mutation leads to postnatal lethality due to constitutive Nrf2 activation. *Nature Genetics*.

[141] Yamamoto M., Kensler T. W., Motohashi H. (2018). The KEAP1-NRF2 system: a thiol-based sensor-effector apparatus for maintaining redox homeostasis. *Physiological Reviews*.

[142] Al-Mubarak B. R., Bell K. F., Chowdhry S. (2021). Non-canonical Keap1-independent activation of Nrf2 in astrocytes by mild oxidative stress. *Redox Biology*.

[143] Wu G. D., Li Z. H., Li X., Zheng T., Zhang D. K. (2020). microRNA-592 blockade inhibits oxidative stress injury in Alzheimer's disease astrocytes *via* the KIAA0319-mediated Keap1/Nrf2/ARE signaling pathway. *Experimental Neurology*.

[144] He P., Yan S., Wen X. (2019). Eriodictyol alleviates lipopolysaccharide-triggered oxidative stress and synaptic dysfunctions in BV-2 microglial cells and mouse brain. *Journal of Cellular Biochemistry*.

[145] Ren X., Yu J., Guo L., Ma H. (2020). TRIM16 protects from OGD/R-induced oxidative stress in cultured hippocampal neurons by enhancing Nrf2/ARE antioxidant signaling via downregulation of Keap1. *Experimental Cell Research*.

[146] Wang X., Wang F., Mao G. H. (2022). NADPH is superior to NADH or edaravone in ameliorating metabolic disturbance and brain injury in ischemic stroke. *Acta Pharmacologica Sinica*.

[147] Bertoni A., Giuliano P., Galgani M. (2011). Early and Late Events Induced by PolyQ-expanded Proteins:. *The Journal of Biological Chemistry*.

[148] Dominah G. A., McMinimy R., Kallon S., Kwakye G. F. (2017). Acute exposure to chlorpyrifos caused NADPH oxidase mediated oxidative stress and neurotoxicity in a striatal cell model of Huntington's disease. *Neurotoxicology (Park Forest South)*.

[149] Kwakye G. F., Jiménez J. A., Thomas M. G. (2019). Heterozygous huntingtin promotes cadmium neurotoxicity and neurodegeneration in striatal cells via altered metal transport and protein kinase C delta dependent oxidative stress and apoptosis signaling mechanisms. *Neurotoxicology*.

[150] Schiavone S., Tucci P., Trabace L., Morgese M. G. (2019). Early celastrol administration prevents ketamine-induced psychotic-like behavioral dysfunctions, oxidative stress and IL-10 reduction in the cerebellum of adult mice. *Molecules*.

[151] Barodia S. K., Creed R. B., Goldberg M. S. (2017). Parkin and PINK1 functions in oxidative stress and neurodegeneration. *Brain Research Bulletin*.

The article "Targeting Molecular Mediators of Ferroptosis and Oxidative Stress for Neurological Disorders" was published in 2022. Journal: Oxid Med Cell Longev.

[152] Maher P., van Leyen K., Dey P. N., Honrath B., Dolga A., Methner A. (2018). The role of Ca^2+^ in cell death caused by oxidative glutamate toxicity and ferroptosis. *Cell Calcium*.

[153] Sun D., Chen X., Gu G., Wang J., Zhang J. (2017). Potential roles of mitochondria-associated ER membranes (MAMs) in traumatic brain injury. *Cellular and Molecular Neurobiology*.

[154] Hayashi T., Su T. P. (2007). Sigma-1 receptor chaperones at the ER-mitochondrion interface regulate Ca(2+) signaling and cell survival. *Cell*.

[155] Kim Y., Jang H. H. (2019). Role of cytosolic 2-Cys Prx1 and Prx2 in redox signaling. *Antioxidants*.

[156] Li L., Acioglu C., Heary R. F., Elkabes S. (2021). Role of astroglial toll-like receptors (TLRs) in central nervous system infections, injury and neurodegenerative diseases. *Brain, Behavior, and Immunity*.

[157] Anfinogenova N. D., Quinn M. T., Schepetkin I. A., Atochin D. N. (2020). Alarmins and c-Jun N-terminal kinase (JNK) signaling in Neuroinflammation. *Cell*.

[158] Samuni Y., Goldstein S., Dean O. M., Berk M. (2013). The chemistry and biological activities of N-acetylcysteine. *Biochimica et Biophysica Acta (BBA) - General Subjects*.

[159] Rushworth G. F., Megson I. L. (2014). Existing and potential therapeutic uses for N-acetylcysteine: the need for conversion to intracellular glutathione for antioxidant benefits. *Pharmacology & Therapeutics*.

[160] Aldini G., Altomare A., Baron G. (2018). N-Acetylcysteine as an antioxidant and disulphide breaking agent: the reasons why. *Free Radical Research*.

[161] Tardiolo G., Bramanti P., Mazzon E. (2018). Overview on the effects of N-acetylcysteine in neurodegenerative diseases. *Molecules*.

[162] Zipfel G. J., Babcock D. J., Lee J. M., Choi D. W. (2000). Neuronal apoptosis after CNS injury: the roles of glutamate and calcium. *Journal of Neurotrauma*.

[163] Baker D. A., McFarland K., Lake R. W. (2003). Neuroadaptations in cystine-glutamate exchange underlie cocaine relapse. *Nature Neuroscience*.

[164] Bridges R. J., Natale N. R., Patel S. A. (2012). System xc- cystine/glutamate antiporter: an update on molecular pharmacology and roles within the CNS. *British Journal of Pharmacology*.

[165] Spencer S., Kalivas P. W. (2017). Glutamate transport: a new bench to bedside mechanism for treating drug abuse. *The International Journal of Neuropsychopharmacology*.

[166] Chen G., Shi J., Hu Z., Hang C. (2008). Inhibitory effect on cerebral inflammatory response following traumatic brain injury in rats: a potential neuroprotective mechanism of N-acetylcysteine. *Mediators of Inflammation*.

The article "Targeting Molecular Mediators of Ferroptosis and Oxidative Stress for Neurological Disorders" was published in 2022. Journal: Oxid Med Cell Longev.

[167] Senol N., Naziroglu M., Yuruker V. (2014). N-acetylcysteine and selenium modulate oxidative stress, antioxidant vitamin and cytokine values in traumatic brain injury-induced rats. *Neurochemical Research*.

[168] Xiong Y., Peterson P. L., Lee C. P. (1999). Effect of N-acetylcysteine on mitochondrial function following traumatic brain injury in rats. *Journal of Neurotrauma*.

[169] Hoffer M. E., Balaban C., Slade M. D., Tsao J. W., Hoffer B. (2013). Amelioration of acute sequelae of blast induced mild traumatic brain injury by N-acetyl cysteine: a double-blind, placebo controlled study. *PLoS One*.

[170] Kyyriäinen J., Kajevu N., Bañuelos I. (2021). Targeting oxidative stress with antioxidant duotherapy after experimental traumatic brain injury. *International Journal of Molecular Sciences*.

[171] Pauletti A., Terrone G., Shekh-Ahmad T. (2019). Targeting oxidative stress improves disease outcomes in a rat model of acquired epilepsy. *Brain*.

[172] Kalish B. T., Whalen M. J. (2016). *Weight drop models in traumatic brain injury*.

[173] Ho M., Yen C. H., Hsieh T. H. (2021). CCL5 via GPX1 activation protects hippocampal memory function after mild traumatic brain injury. *Redox Biology*.

[174] Mahumane G. D., Kumar P., Pillay V., Choonara Y. E. (2020). Repositioning N-acetylcysteine (NAC): NAC-loaded electrospun drug delivery scaffolding for potential neural tissue engineering application. *Pharmaceutics*.

[175] Sharma A., Liaw K., Sharma R., Zhang Z., Kannan S., Kannan R. M. (2018). Targeting mitochondrial dysfunction and oxidative stress in activated microglia using dendrimer-based therapeutics. *Theranostics*.

[176] Jhelum P., Santos-Nogueira E., Teo W. (2020). Ferroptosis mediates cuprizone-induced loss of oligodendrocytes and demyelination. *The Journal of Neuroscience*.

[177] Kenny E. M., Fidan E., Yang Q. (2019). Ferroptosis contributes to neuronal death and functional outcome after traumatic brain injury. *Critical Care Medicine*.

[178] Chen J., Yang L., Geng L. (2021). Inhibition of acyl-CoA synthetase long-chain family member 4 facilitates neurological recovery after stroke by regulation ferroptosis. *Frontiers in Cellular Neuroscience*.

[179] Hao L., Mi J., Song L. (2021). SLC40A1 mediates ferroptosis and cognitive dysfunction in type 1 diabetes. *Neuroscience*.

[180] Do Van B., Gouel F., Jonneaux A. (2016). Ferroptosis, a newly characterized form of cell death in Parkinson's disease that is regulated by PKC. *Neurobiology of Disease*.

[181] Xie Y., Hou W., Song X. (2016). Ferroptosis: process and function. *Cell Death and Differentiation*.

